# Imaging Characteristics of Invasive Pulmonary Fungal Infection Secondary to Hematological Diseases and Comparison before and after Treatment

**DOI:** 10.1155/2021/3736108

**Published:** 2021-09-29

**Authors:** Jun-Wei Wang, Fang-Fang Yang, Chuan-Yu Zhang, Ji-Zheng Lin, He-Xiang Wang, Wen-Jian Xu

**Affiliations:** ^1^Department of Radiology, The Affiliated Hospital of Qingdao University, No. 16 Jiangsu Road, Qingdao 266001, Shandong, China; ^2^Department of Nephrology, The Affiliated Hospital of Qingdao University, No. 16 Jiangsu Road, Qingdao 266001, Shandong, China

## Abstract

Fungal infections have become crucial factors that threaten the prognosis and survival of blood disease patients. Here, we aim to analyze the epidemiological characteristics and early and advanced CT (computed tomography) manifestations of patients with invasive pulmonary fungal infections secondary to blood system diseases. 65 hospitalized patients from October 2018 to October 2020 with invasive pulmonary fungal infections secondary to blood diseases were enrolled. Blood diseases were recorded according to clinical and imaging data, and the serum galactomannan test (GM test) was conducted. Two senior radiologists analyzed the CT data and recorded the distribution of the lesions and CT signs. We analyzed and counted the first chest CT scan images of patients with nodule/mass type secondary to hematological diseases and invasive pulmonary fungal infection. The first CT nodules or mass-type lesions were statistically significant in nodule size, the number of lesions, distribution, and accompanying signs. Pulmonary fungal infection was common in both lungs during 7-day, 14-day, and 30-day follow-up CT. We also found that the nodular mass type was the main manifestation in the positive group of the GM test. Both the positive group and the negative group had the highest incidence of nodules. The incidence of air crescent signs in nodules or mass lesions in the positive group was higher than in the negative group, and the difference was statistically significant. To conclude, follow-up CT signs after antifungal treatment were highly sensitive to the early diagnosis of hematological diseases and secondary invasive pulmonary Eumycetes infection, which could be used for clinical treatment to provide help. GM test results were also related to CT manifestations such as air crescent sign, cavity, and halo sign.

## 1. Introduction

Hematological diseases, such as leukemia, lymphoma, severe aplastic anemia (SAA), and hematopoietic stem cell transplantation (HSCT), are prone to secondary blood system abnormalities caused by bone marrow transplantation or immunocompromised stage and other diseases [1]. Deep fungal infections and secondary fungal infections have become important factors affecting the prognosis and survival of blood disease patients [2]. However, due to the existence of underlying diseases, the condition is more complicated, and its imaging manifestations are diverse and overlap each other [3]. The author focuses on reviewing the status quo of imaging studies of pulmonary fungal infections secondary to blood diseases. The incidence of deep fungal diseases has risen sharply in the past two centuries. A survey of 115 hospitals in the United States showed that the fungal infection rate in the 1990s was 1.9 times that of the 1980s. Another scholar reported that the incidence of fungal infection in 2004 was 214 times that of the 1990s. Yamazaki et al. reported that the incidence of fungi in patients with acute myeloid leukemia (AML), acute lymphocytic leukemia (ALL), chronic myelogenous leukemia, myelodysplastic syndrome (MDS), and lymphoma (NHL) was, respectively, 35.4%, 43.6%, 42.8%, 22.2%, and 10.5%. Therefore, the problem of blood system diseases combined with fungal infections should arouse great attention. As far as lung pathogenic bacteria are concerned, *Candida*, especially *Candida albicans*, is the main lung pathogenic fungus. However, in recent years, the infection rate of *Candida albicans* has declined, and the infection rate of non-*Candida albicans* has increased. Pathogenic bacteria include *Aspergillus*, *Cryptococcus*, and *Mucor* [4].

Fungi can be divided into pathogenic fungi and conditional pathogenic fungi. Most of the pathogens of deep fungal infection are conditional pathogens, which can cause disseminated system infection when the body's immunity is reduced. The main reasons why patients with hematological diseases are susceptible to fungus infection can be roughly summarized as follows. (1) Changes in blood composition of patients with hematological malignancies reduce the quality and quantity of lymphocytes and neutrophils and weaken the body's immunity. (2) High-dose chemotherapy, radiotherapy, and immunosuppressive therapy have further deepened the immune dysfunction of the body, resulting in prolonged neutropenia and deficiency. (3) Patients with hematological malignancies use a wide variety of antibiotics, large doses, long treatment courses, broad antibacterial spectrum, frequent replacements, and multiple combination medications, leading to the disappearance of the antagonistic antibacterial group in the normal flora of the body. (4) The application of adrenal cortex hormones further weakens the patient's anti-infection ability. According to research conducted by the Department of Imaging Diagnostics, it is believed that fungal infections are most likely to occur during the two courses of chemotherapy. The chance of improving immune function in the third to fifth courses of chemotherapy is low. After the sixth course of treatment, hematopoietic function and immune function are further reduced and the chance of fungal infection increases again. In addition, the incidence of high-dose chemotherapy, neutropenia, elderly patients, use of broad-spectrum antibiotics and high-dose glucocorticoids, failed graft implantation, and the previous history of fungal infection or organ dysfunction is high and serious. When the host's functional barrier is destroyed or foreign objects enter, it is susceptible to *Candida* infection. Granulocyte dysfunction is a high-risk factor for fungal diseases such as *Aspergillus, Candida*, and *Mucor*, while those with cellular immune suppression are susceptible to candidiasis and zygosity disease, coccidioidomycosis, cryptococcosis, histoplasmosis, etc. [5].

The main clinical features of hematological diseases with fungal infections are the following. (1) Fever: as blood diseases themselves can also cause fever, fungal infections are easily confused; in some patients who are treated with high-dose hormone therapy, fever caused by latent fungal infection is often covered by hormone therapy. (2) Respiratory symptoms: there may be fever, cough, sputum expectoration, and other symptoms. Some patients have hemoptysis, fatigue, weight loss, chest pain, and dyspnea. There is no significant difference between common bacterial infections and other diseases. In special populations, such as patients with hematopoietic stem cell transplantation, some rare clinical symptoms may occur, such as diffuse lung injury caused by the invasive fungal infection of the lung, pulmonary fibrosis, clinical manifestations of interstitial pneumonia syndrome, and severe cases that can be life-threatening. But different strains have different imaging manifestations at different stages of the disease. Although characteristic manifestations such as the air-half-moon sign or CT halo sign are sometimes seen, the imaging findings of opportunistic fungal infections, especially fungal infections secondary to blood diseases, are generally not characteristic and are associated with other lung diseases and even lung cancer. There will be overlaps in performance. *Candida* infection: gross specimens often show the symmetrical distribution of bleeding nodules in both lungs. The change under a light microscope is a microabscess. After the pseudohyphae grow into the capillaries, arterioles, and arterioles, they continue to penetrate the lung tissues and airways surrounding the blood vessels. Subpleural nodules and necrotizing vasculitis can be seen. Pulmonary embolism can occur when the middle and small arteries of the lung are completely blocked by *Candida* spores and pseudohyphae. The most common manifestation of imaging is patchy infiltrates of the lung interstitium and alveoli, involving both lung fields and rarely the lung apex. The shadow often changes during the disease course. Multifocal consolidation has no prevalent sites. Pathologically, it is bronchopneumonia, alveolar hemorrhage, and exudation; alveolar edema, diffuse alveolar septum, and hyaline membrane thickening. Abnormal chest radiographs include patchy consolidation of the lower lung, with less diffuse grid or grid nodular lesions.

Due to the risks of fungus and the complexity of blood diseases, this kind of infection was difficult to be monitored, evaluated, and treated. Currently, the lack of research that concentrated on this area and the lack of connection between the CT signs, fungal infection, and blood diseases were the motivation of our study. Therefore, we planned to analyze the characteristics and early and advanced CT manifestations of patients with invasive pulmonary fungal infections secondary to blood system diseases.  Section 1 discussed the introduction, Section 2 described the method and materials, Section 3 showed the results and main findings, and Section 4 discussed our results.

## 2. Materials and Methods

### 2.1. General Information

We used a retrospective collection of 65 hospitalized patients (35 males and 30 females, middle-age: 40 years old) with hematological diseases diagnosed or clinically diagnosed or suspected of pulmonary fungal infection from October 2018 to October 2020 in our hospital as the research objects, whose clinical data, laboratory examinations, and images were recorded. Scientific data, including name, gender, age, underlying disease, clinical manifestations, first chest CT signs of pulmonary fungal infection, recheck CT time and signs, and results of the galactomannan test (GM test) during the same period (chest CT scan ±2 days on the day of inspection), were also collected. Inclusion criteria were the following: (1) refer to my country's 2010 “Diagnosis Criteria and Treatment Principles of Invasive Fungal Infection in Patients with Hematological Diseases/Malignant Tumors (Third Revision)” and 2014 “Diagnosis of Invasive Mycosis in Patients with Hematological Diseases/Malignant Tumors Interpretation of Standards and Treatment Principles (Fourth Revised Edition)” established diagnostic criteria: (1) patients with immunodeficiency such as neutrophils below O. 5x109/L patients and patients with hematological malignancies; (2) patients who have complete clinical data and imaging data. The objects were divided into confirmed IPFI, clinically diagnosed IPFI, and proposed IPFI. (1) The confirmed IPFh meets at least 1 host factor, 1 clinical criterion or 2 secondary clinical features, and 1 microbiology (lung tissue specimen, sterile specimen (bronchoalveolar lavage fluid, sputum), and positive blood culture) or histopathological basis; (2) clinical diagnosis of IPFI meets at least 1 host factor, 1 clinical standard, and 1 basis of microbiological examination; (3) the proposed IPFI at least meets 1 host factor, 1 clinical standard, and lack of microbiological standards. Exclusion criteria were the following: (1) patients with bronchopulmonary fungal infection caused by fungal parasitism and allergies; (2) patients with concurrent infections of other pathogens (such as bacteria, mycoplasma, viruses, and current tuberculosis infection).

### 2.2. Instrument and Equipment

Using Somatom Sensation dual-source spiral CT machine and Somatom Sensation 64-slice spiral CT machine, the patient takes a breath-hold scan in the supine position to perform a routine exposure dose scan of the whole lung. The reconstruction layer thickness and interval are 3 mm, respectively. The scanning range includes the lung tip to the costophrenic angle. Layer thickness and layer spacing are 3 mm, respectively, using B3If. The B80f algorithm performs reconstruction. The contrast-enhancing agent was iodophor, and intravenous injection was with a high-pressure syringe. The injection speed was 3.0–3.5 ml/s. The injection dose was 80.85 ml. The arterial phase was scanned for 30 seconds, and the arterial phase was scanned for 30 seconds after the end of the venous phase, using Dana Biological Aspergillus galactomannan quantitative detection kit (ELISA method).

### 2.3. CT Image Analysis

Two senior chest radiology specialists read the pictures separately and analyzed the chest CT image data before and closest to the diagnosis of the patient. When there is a disagreement, a consensus is reached after consultation. The main lesions evaluated include nodules (small nodules are less than 1 cm in diameter, while large nodules are 1 cm–3 cm in diameter), masses (more than 3 cm in diameter), consolidation, ground-glass shadow, mesh shadow, bronchial vascular bundle thickening, pleural effusion, hilar and mediastinal lymph nodes, enlarged or multiple different types of lesions appearing in the same CT scan image called mixed lesions, and only one type of lesions appearing in the same CT scan image called simple lesions. The evaluation content of various types of lesions includes the distribution of nodules and masses (lobular center, tree bud sign, around the bronchial vascular bundle, and subpleural), number (single, multiple including 2–10, or more than 10), multiple nodules segments which are divided into clustered type (limited to a single lung lobe) and scattered distribution type (distributed in multiple lung lobes), size (less than 1 cm, 1 cm–3 cm, and greater than 1 cm), edge (halo sign), the internal structure (cavity, air-half-moon sign), distribution of consolidation (subpleural, around the bronchial vascular bundle, lobular type, and nonlobular type), number (single or multiple), the internal structure (cavity, air-half-moon sign), and distribution of ground-glass shadow (focal, segmental, and diffuse); with the tracheal carina as the boundary, the aforementioned lesions are divided into the main area of the upper lung (above the tracheal carina) and the main area of the lower lung (below the tracheal carina). The main peripheral zone and the main internal zone (the line between the tracheal carina and the midpoint of the parietal pleura is the boundary) are randomly distributed. Hilar and mediastinal lymphadenopathy is defined as a single or multiple lymph nodes with a short diameter exceeding 1 cm. After evaluating the CT findings of pulmonary cryptococcosis, it is divided into the following four types according to the nature and distribution characteristics of the main lesions: single nodule or mass type, multiple clustered nodules, multiple scattered nodules, and bronchopneumonia type.

### 2.4. Statistical Analysis

The data was collected and imported to SPSS16.0 software which was commonly used statistical software and then analyzed. The absolute number was expressed as mean ± standard deviation, the relative number was expressed as rate and ratio, and the comparison between groups was analyzed by *χ*^2^ or Fisher's exact probability method. *P* < 0.05 indicated a significant difference.

## 3. Results

### 3.1. First CT Distribution of Patients with Invasive Pulmonary Fungal Infection Secondary to Blood System Diseases

In 65 patients with invasive pulmonary fungal infection secondary to hematological diseases, the first chest CT scan was performed, and the CT image signs were recorded in two major types, namely, the nodule type (the CT signs are simple nodules or masses) and mixed type (CT signs include two or more), for statistics. There were 40 cases of nodule/mass type and 25 cases of mixed type, including 2 cases of ground glass, 9 cases of atelectasis, 7 cases of interstitial inflammation, and 7 cases of tree bud sign. Analyze the two types of data, record the incidence of lesions, and perform statistical analysis. The first CT signs have a high incidence of nodules/mass, as shown in Table 1.

### 3.2. The First CT Signs of Nodule/Mass-Type Lesions Secondary to Invasive Pulmonary Fungal Infection of Blood System Diseases

Analysis and statistics of the first chest CT scan of patients with invasive pulmonary fungal infections secondary to hematological diseases with nodule/mass type revealed 40 cases of nodule/mass type, 394 lesions, 114 of which are micronodules. There were 146 nodules, 119 nodules, and 15 masses. The first CT nodules or mass type lesions were statistically significant in nodule size, the number of lesions, distribution, and accompanying signs (cavity, air crescent sign, and halo sign). See Table 2 and Figure 1 for details.

### 3.3. Follow-Up Results

65 patients underwent CT follow-up examinations ranging from 1 to 10 times after the diagnosis of pulmonary fungal infection, and the follow-up period ranged from 2 days to 200 days. The first CT results showed 9 patients with a unilateral single disease and 6 patients with unilateral multiple diseases. There were 27 more cases, and the number of infections increased with the prolonged follow-up time. Pulmonary fungal infection is common in both lungs during 7-day, 14-day, and 30-day CT follow-up. For details, see Tables 3 and 4.

### 3.4. Serum GM Test and First CT Findings

In 65 patients with invasive pulmonary fungal infections secondary to hematological diseases, 25 were examined by blood galactomannan test (GM test) for the first time: 17 cases were positive in GM test (≥0.85 ug/L) and 8 was negative in the *G* test example. The GM antigen test has been widely used to diagnose invasive pulmonary aspergillosis [6]. Serum GM test was positive in 18 cases and negative in 9 cases during the 7-day follow-up. On the 14th day, the serum GM test was positive in 17 cases and negative in 10 cases. The 30-day serum GM test was positive in 25 cases and negative in 5 cases.  Table 5 shows that the nodular mass type was the main manifestation in the positive group of the GM test. Both the positive group and the negative group had the highest incidence of nodules with a diameter of 5.10 mm. The incidence of air crescent signs in nodules or mass lesions in the positive group was higher than that in the negative group. The difference was statistically significant (*P* = 0.012); see details in Tables 6 and 5.

## 4. Discussion

Pulmonary infection has always been one of the main diseases threatening human health. In the 1990s, deaths caused by infectious diseases accounted for one-third of the global deaths, and lung infections ranked first among all types of infections. With the development of organ transplantation, the widespread application of tumor radiotherapy and chemotherapy technology and immunosuppressive agents, and the increasing number of Acquired Immune Deficiency Syndrome (AIDS) patients, population-immunocompromised host (ICH) may have one or more links of immunodeficiency, and different types of immunodeficiency and duration lead to different susceptibility to pathogens. For example, when the duration of granulocytopenia or deficiency is less than 3 weeks, the risk of bacterial infection is significantly increased; greater than 3 weeks, the risk of fungal infection is significantly increased, while humoral immune deficiency and complement deficiency are prone to infection by capsular bacteria [7]. In this case, the incidence of invasive fungal infections, especially IPFI, has been increasing year by year and has become a research focus in recent years.

A survey of fungal infections in 115 hospitals in the United States showed that the rate of invasive fungal infections in hospitalized patients in the 1990s was 1.9 times that of the 1980s. The survey results in 2004 showed that the fungal infection rate was 2.4 times that of the 1990s [8]. The incidence of invasive fungal infections calculated by Peking Union Medical College Hospital in 2003 was 3.6 times that of the 1990s. Invasive fungal diseases mostly occur in patients with serious underlying diseases, with poor prognosis and high mortality. The mortality rate of candidiasis can reach 40%. The incidence of invasive aspergillosis in kidney transplantation, liver transplantation, bone marrow transplantation, and lung transplantation patients is 1%, 2%, 7%, and 9%, respectively, and the average mortality rate is as high as 55 to 92%, which is the main cause of death in 10 to 15% of transplant patients [9]. Early detection and diagnosis of pulmonary fungal infections, especially IPFI, so that timely and effective antifungal treatment can be performed, are key to treating pulmonary fungal infections and reducing mortality. The gold standard for the diagnosis of deep fungal infection is the pathogenic diagnosis, and sputum smear or culture is the most commonly used method for the diagnosis of lung fungal infection. Although some patients with pulmonary fungal infection can find pathogens from smears, sputum specimens are easily contaminated by oral secretions, and the false positive rate is high; fungal culture takes a long time, and earlier positive results could be obtained from only 3.2% of patients [10]. Lin et al. have reviewed the epidemiology of the invasive fungal disease in patients with hematological diseases [11] and pointed out that the secondary fungal infection was one of the main factors leading to the death of patients with hematological diseases. Currently, the monitoring of fungal infections mostly relied on the results of laboratory examinations but ignored the damage of fungus on the lungs of patients. CT scan could remedy this situation [12].

Due to the atypical symptoms and the delay of laboratory examinations, IPFI is sometimes difficult to distinguish from common bacterial lung infections [13], especially for immunosuppressive hosts such as organ transplants and malignant tumors. IPFI is seriously ill with symptoms, signs, and laboratory. The examination lacks specificity and is often concealed by the underlying disease or the drugs used, making it difficult to identify [14]. Routine blood culture is also very insensitive. The positive rate of blood culture in patients with invasive *Candida* pneumonia confirmed by autopsy is less than 50% [15]. Even with the newer diagnostic methods, such as hemolytic precipitation and culture of *Candida*, the positive rate is not high enough. However, serological methods for the diagnosis of *Candida* antigens or antibodies are not perfect and popular. With the application of invasive biopsy techniques such as bronchoscopy and lung puncture, the diagnosis rate of IPFI has increased. Fine-needle aspiration biopsy can diagnose 50–67% of IPFI, but the overall incidence of complications is 15%. And it is higher in patients with platelet counts below 30,000/mm^3^ [16].

Therefore, looking for a fast, reliable, safe, and convenient method for diagnosing pulmonary fungal infection has great application value and important practical significance for early detection of the disease, timely treatment, and reduction of mortality. The development of imaging science, especially the continuous innovation of thin-slice spiral CT imaging technology, has made it possible to clearly show the fine structure and microscopic pathological changes of the lungs. The early detection and diagnosis of pulmonary fungal infections by imaging methods are an important subject of current research in this field. Affected by the patient's immune status, the types and quantities of invading pathogens, and the route of infection, the imaging manifestations of pulmonary fungal infections are very complicated. At present, there are not many imaging studies on the disease, and the findings have practical value for the diagnosis of IPFI few characteristic signs. The 2006 “Diagnostic Criteria and Treatment Principles of Invasive Pulmonary Fungal Infection” listed the characteristic imaging manifestations of invasive pulmonary *Aspergillus* infection and pneumocystis pneumonia as the main clinical indicators of the diagnostic criteria [17], but other characteristic imaging findings of IPFI have not yet been clarified. The imaging misdiagnosis is 64.29% [18], which can be misdiagnosed as bronchitis, bacterial pneumonia, lung cancer, tuberculosis, and metastatic lung cancer.

In this study, 65 patients with invasive pulmonary fungal infections secondary to hematological diseases were scanned for the first chest CT scan, and the CT image signs were recorded in two major types, namely, the nodule type (the CT signs are simple nodules), mass, and mixed type (CT signs contain two or more than two types), for statistics. There were 40 cases of nodule/mass type and 25 cases of mixed type, including 2 cases of ground glass, 9 cases of atelectasis, 7 cases of interstitial inflammation, and 7 cases of tree bud sign. Analyze the two types of data, record the incidence of lesions, and perform statistical analysis. The first CT signs have a high incidence of nodules/mass. Analyze and count the first chest CT scan images of patients with nodule/mass type secondary to hematological diseases and invasive pulmonary fungal infection. There are 40 cases of nodule/mass type with a total of 394 lesions, of which 114 are micronodules. There were 146 nodules, 119 nodules, and 15 masses. The first CT nodules or mass type lesions were statistically significant in nodule size, the number of lesions, distribution, and accompanying signs (cavity, air crescent sign, and halo sign). 65 patients underwent CT follow-up examinations ranging from 1 to 10 times after the diagnosis of pulmonary fungal infection, and the follow-up period ranged from 2 days to 200 days. The first CT results showed 9 patients with unilateral single disease and 6 patients with unilateral multiple diseases. There were 27 more cases, and the number of infections increased with the prolonged follow-up time. Pulmonary fungal infection was common in both lungs during 7-day, 14-day, and 30-day follow-up CT. In 65 patients with invasive pulmonary fungal infections secondary to hematological diseases, 25 were examined by blood galactomannan test (GM test) for the first time, 17 cases were positive in GM test (≥0.85ug/L), and 8 was negative in the *G* test example. Serum GM test was positive in 18 cases and negative in 9 cases during the 7-day follow-up. On the 14th day, the serum GM test was positive in 17 cases and negative in 10 cases. The 30-day serum GM test was positive in 25 cases and negative in 5 cases.  Table 5 shows that the nodular mass type was the main manifestation in the positive group of the GM test. Both the positive group and the negative group had the highest incidence of nodules with a diameter of 5.10 mm. The incidence of air crescent signs in nodules or mass lesions in the positive group was higher than that in the negative group, and the difference was statistically significant.

In summary, the first CT signs and follow-up CT signs of invasive pulmonary fungal infection secondary to blood system diseases are highly sensitive to the early diagnosis of blood disease pulmonary fungal infection, which can provide help for clinical treatment. The distribution of lesions, the size and number of nodules, and whether they are accompanied by cavities, air crescent sign, tree bud sign, halo sign, and the antihalo sign can provide help in the diagnosis and differential diagnosis of invasive lung fungal infection. CT scan accurately assessed the efficacy of antifungal therapy before and after the treatment and on follow-up studies.

## 5. Conclusion

Follow-up CT signs after antifungal treatment are highly sensitive to the early diagnosis of invasive lung fungal infections secondary to hematological diseases and can provide help for clinical treatment. The combined detection of the GM test improves the sensitivity of the test, and the continuous follow-up of GM test value changes has certain clinical significance for the early diagnosis of invasive lung fungal infection. The results of the first GM test are related to the first CT signs, such as the number of lesions, air crescent sign, cavity, and halo sign. In the future, we will continuously collect more clinical data and try to evaluate the effectiveness of antifungal drugs using CT images to provide new insights for the therapeutic strategies against lung fungal infection.

## Figures and Tables

**Figure 1:** Case: a patient with acute lymphoblastic leukemia and pulmonary *Aspergillus* infection. The first CT showed multiple lung nodules with crescent sign formation in right lung lesions (a). After antifungal treatment, a 7-day follow-up CT showed cavities and consolidation in the right lung nodules and left lung fibrous lesions (b). The 14-day follow-up showed that CT right lung nodules disappeared, cavities increased, and left lung fibrous foci existed (c). The 30-day follow-up CT showed that the right lung cavity was reduced, and the left lung fibrous foci existed (d).

**Table 1:** The first CT signs of patients with invasive pulmonary fungal infection secondary to blood system diseases.

CT signs	Number of cases (*n*)	Incidence (%)
Simple	40	61.54
Nodules/lumps	40	61.54
Hybrid	25	38.46
Atelectasis	9	13.85
Interstitial inflammation	7	10.77
Tree bud sign	7	10.77
Ground glass	2	3.08

**Table 2:** Primary CT lesion size and accompanying signs of simple-type secondary invasive lung fungal infection of hematological diseases.

Nodule size	Tiny nodules (<5 mm)	Small nodules (5–10 mm)	Nodules (10–30 mm)	Lumps (>30 mm)	*P* value
Proportion	114	146	119	15	
Halo sign	3	45	46	10	≤0.001
Hollow	2	8	19	11	≤0.001
Air crescent sign	1	3	25	11	≤0.001

**Table 3:** Comparison of lesion distribution in CT follow-up of invasive pulmonary fungal infection secondary to hematological diseases.

Unilateral distribution	First CT	7 D	14 D	30 D
Single-side single-shot	9	8	6	6
Multiple shots on one side	6	10	8	11
Bilateral multiple	27	30	28	28

**Table 4:** Follow-up comparison of CT signs of invasive pulmonary fungal infections secondary to hematological diseases.

Time	Number of cases	Hollow (%)	Air crescent sign (%)	Halo sign (%)
First	45	9.50	0.00	24.65
7 D	42	10.23	13.26	18.59
14 D	33	21.36	3.72	21.56
30 D	33	17.98	14.36	3.54
*X* ^2^		1.95	2.65	6.58
*P* value		0.115	0.063	0.035

**Table 5:** Changes in the number of patients in the follow-up GM test.

GM trial	First	7 D	14 D	30 D
Positive	25	19	16	15
Negative	5	11	14	15
*P* value	0.03	0.05	0.58	1.00

**Table 6:** GM test and first CT performance and *P* value.

CT sign	GM trial (−) *n* = 8	GM trial (+) *n* = 17	*P* value
Nodular mass	8	17	
<5 mm	1	4	0.523
5–10 mm	5	10	0.568
10–30 mm	1	2	0.689
≥30 mm	1	1	0.581
Hollow	0	1	0.791
Air crescent sign	0	3	0.013
Halo sign	0	13	0.789
Consolidation	0	6	0.269
Pleural effusion	0	2	0.548

## Data Availability

The simulation experiment data used to support the findings of this study are available from the corresponding author upon request.
